# Prediction of Sacral Screw Loosening after Lumbosacral Surgeries Involving Rigid Fixation of Sacral Bone Using Preoperative Computed Tomography Scans

**DOI:** 10.1155/2022/7123139

**Published:** 2022-05-23

**Authors:** Aikeremujiang Muheremu, Maihemuti Yakufu, Junyao Jiang, Muradil Mardan, Lei Li, Rui Zhang, Abudunaibi Aili, Zhaohui Luo

**Affiliations:** ^1^Department of Spine Surgery, Sixth Affiliated Hospital of Xinjiang Medical University, 39, Wuxing Nan Rd, Tianshan District, Urumqi, Xinjiang 86830001, China; ^2^Department of Orthopaedics, Sixth Affiliated Hospital of Xinjiang Medical University, 39 Wuxing Nan Rd, Tianshan District, Urumqi, Xinjiang 86830001, China; ^3^Class of 1806 Clinical Medicine, School of Basic Medical Sciences, Henan University of Science and Technology, 263 Kaiyuan Avenue, Luolong District, Luoyang, Henan 86471023, China; ^4^Department of Clinical Medicine, Medical College of Tongji University, 50 Chifeng Rd, Yangpu District, Shanghai 200092, China; ^5^Department of Radiology, Sixth Affiliated Hospital of Xinjiang Medical University, 39 Wuxing Nan Rd, Tianshan District, Urumqi, Xinjiang 86830001, China; ^6^Department of Nursing, Sixth Affiliated Hospital of Xinjiang Medical University, 39 Wuxing Nan Rd, Tianshan District, Urumqi, Xinjiang 86830001, China

## Abstract

**Objective:**

To find a preoperative computed tomography-based method to predict the incidence of sacral screw loosening and assist surgical planning.

**Methods:**

Surgically treated patients for degenerative lumbosacral disorders with rigid pedicle screw fixation of patients with L5-S1 vertebra in our center from January 2016 to January 2021 were retrospectively included in the current study. CT scan attenuation of the horizontal plane of the sacrum was measured with Hounsfield units (HU). Postoperative X-ray tests were used to diagnose screw loosening. The data was analyzed by independent sample *t*-tests, *X*^2^ analysis, Pearson correlation analysis, and ROC curve analysis.

**Results:**

A total of 162 (114 male, 48 female, average age 63.7 ± 7.3 years) patients were included in the final analysis. Significant differences were found between the screw loosening group and nonloosening group concerning the HU value of the sacrum at the horizontal plane (*P* < 0.01). In ROC curve analysis, AUC was 0.674 (95% CI: 0.592-0.756). A cutoff of 200 HU provided 64.8% sensitivity and 62.4% specificity, and a cutoff of 150 HU provided 90.2% sensitivity.

**Conclusions:**

Analyzing 162 patients with at least 12 months of follow-up, we propose cutoff CT attenuation values of 200 HU and 150 HU to take moderate and radical measures of screw augmentation to prevent screw loosening in the sacral bone.

## 1. Introduction

In lumbar spinal stenosis, lumbar spondylolisthesis, and other lumbosacral degenerative diseases, lumbosacral decompression and pedicle screw fixation are often a necessity [1, 2]. However, due to the special anatomical structure and biomechanical properties of the sacrum, lumbosacral fixation is often followed by complications such as the formation of pseudoarticular joints, loosening, and breakage of pedicle screws. Screw loosening is one of the main complications of rigid fixation in spine surgery. It may lead to undesirable outcomes such as pain and decline of motility and life quality. Reported incidence of sacral pedicle screw loosening in the current literature ranges from 15.6% to 46.5%, which is significantly higher than the incidence of lumbar screw loosening [3–5]. Due to poor bone quality in the elderly population, internal fixation-related complications are especially common in patients with lumbosacral degenerative disorders [6].

At present, techniques commonly used to enhance the strength of the sacral pedicle screw fixation include double and tricortical fixation, application of expanding screws, S1-2 combined screw fixation, iliac screw fixation, and the cement-reinforced screw fixation [7–9]. However, sacral double or tricortical fixation and expanding screw fixation techniques still face certain risk of screw loosening, while S1-2 combined screw fixation and iliac screw fixation may lead to extensive soft tissue damage. Bone cement augmentation technique is easy to carry out and has better fixation strength, but there are concerns that it could cause complications such as fatal pulmonary embolism [10, 11]. Therefore, there is an urgent need for a preoperative measure with high sensitivity to predict screw loosening so as to help the surgeon decide whether or not to apply screw augmentation techniques in a specific patient. Considering that preoperative computed tomography (CT) scans are regularly carried out before spine surgeries, here, we report a computed tomography scan-based method to predict screw loosening in the sacral spine after rigid lumbosacral fixation.

## 2. Materials and Methods

### 2.1. Patient Inclusion and Exclusion

All procedures were approved by the ethical committee of our hospital, and written consent was achieved from patients before treatment. All the procedures were carried out according to the Helsinki declaration. Surgically treated patients for degenerative lumbosacral disorders with bicortical pedicle screw fixation and interbody fusion of the sacral vertebra in our center from January 2016 to January 2021 were retrospectively included in the current study. Other inclusion criteria include the age of 50 years or older, computed tomography scans carried out before and after surgery, followed up for more than 12 months, no previous surgical intervention in the sacral region, and no previous congenital malformations such as congenital scoliosis. Patients with malignant tumor of the spine, previous surgeries at the lumbosacral region, and active inflammation before and after surgery were excluded.

### 2.2. Outcome Assessment

Computed tomography scans were carried out in the department of radiology of our hospital. Patients underwent CT scans (GE 32 row spiral CT, US) before the surgery. Two independent examiners used PACS (GE electrics, US) to measure the HU value. The region of interest (ROI) with a maximum diameter within the cortex of the sacrum was determined on the horizontal plane, and the radiologic attenuation was recorded in HU automatically (Figure 1). CT scan attenuation of the horizontal plane of the sacrum was measured with Hounsfield units (HU). Postoperative anteroposterior X-ray tests were used to diagnose screw loosening. Patient demographic data including patient age, gender, and body mass index (BMI) were recorded in addition to radiological parameters.

Two senior spine surgeons independently evaluated screw loosening and bone fusion by the follow-up X-ray and CT scans. More than 1 mm of clear zone around the screw was used as a reference to diagnose screw loosening [12]. Nonfusion was determined if there was no continued trabecular bone in flexion-extension X-ray film and in cases with more than 3 mm anterior translation and more than 5° rotation.

### 2.3. Statistical Analysis

Demographic characteristics between the two groups were compared with independent sample *t*-tests (measurement data) and *X*^2^ Fisher's exact test analysis (count data). Pearson correlation analysis and ROC curve analysis were used to further evaluate applicability of HU on the prediction of screw loosening. IBMSPSS 24.00 software was used for all statistical analysis. Continuous variables were recorded as mean ± standard deviation. The difference was considered significant when *P* < 0.05.

## 3. Results

A total of 162 (114 male, 48 female, average age 63.7 ± 7.3 years) patients underwent sacral screw fixation in the treatment of lumbosacral spinal disorders during the study period. They were treated for diseases including spondylolisthesis, lumbar spinal stenosis, degenerative scoliosis, and spondylodiscitis. The average time of follow-up was 18.8 ± 11.4 months (range 12-53 months). The average HU value of the sacrum was 212.6 ± 54.3. There were no significant differences between the screw loosening group and non-screw loosening group concerning patient gender, BMI, habit of smoking, and whether or not the patient had diabetes or suffered from spondylolisthesis (*P* > 0.05). The difference was significant between the groups concerning patient age, formation of pseudoarthrosis during follow-up, and HU value of the sacrum at the horizontal plane (*P* < 0.001). The average HU value of sacrum was 225.8 ± 62.4 and 205.6 ± 55.9 in the non-screw loosening group while it was 188.9 ± 54.6 and 166.5 ± 52.5 in the screw loosening group (Table 1).

Pearson correlation analysis on the indicators showed significant correlation between the incidence of screw loosening and the formation of pseudoarthrosis (*P* < 0.01) and HU values measured on the horizontal plane (*P* < 0.01). Although pseudoarthrosis is significantly correlated to the incidence of screw loosening, considering the objective of the current study which was to find a prediction measure for sacral screw loosening, here, we only carried out further analysis on the sacral HU value on different planes. ROC curve analysis was carried out to find the predictive value of computed tomography on screw loosening after sacral screw implantation, and the results revealed that area under the curve (AUC) was 0.674 (95% CI: 0.592-0.756), indicating a higher predictive value of CT attenuation measured on the horizontal plane (Figure 2).

Although ROC curve analysis failed to provide an ideal cutoff HU value with high sensitivity and specificity to predict the incidence of screw loosening, a further look into the statistical data showed that on the horizontal plane, a cutoff of 200 HU provided 64.8% sensitivity and 62.4% specificity, and a cutoff of 150 HU provided 90.2% sensitivity and 20.0% specificity.

## 4. Discussion

Due to the relatively porous structure and large stress load on the sacrum, pedicle screws in the sacral bone are liable to loosening after lumbosacral surgery, especially in elder patients with low bone mineral density [13].

In patients with high probability of screw loosening, it is plausible to use preventive pedicle screw augmentation. Among the various methods of screw augmentation, bone cements and expandable screws are the most tested [14–16]. In the study of Mueller et al. [17], 237 vertebrae in 98 patients were fixed by 474 cement-augmented pedicle screws. Although no symptomatic cement leakage was observed, asymptomatic paravertebral cement leakage was seen in 88 patients and pulmonary cement embolism was found in 4 patients. In the study of Gazzeri et al. [18], 174 expandable screws were used to treat 33 patients with traumatic and degenerative spinal diseases, while 50 patients with similar conditions were treated with conventional screws. The mean ODI score improved from 83.78% to 29.7% after surgery, and no screw loosening was found during a 2-year follow-up in patients treated with expandable screws. When reviewing the current literature, we found that most studies show a significant decrease in the incidence of screw loosening by various techniques such as bicortical fixation, expandable screws, or bone cement augmentation [19–25].

However, screw augmentation techniques are not without their drawbacks. Screw augmentation increases the risk of cement leakage and the incidence of deep tissue infection, operative time, and cost of treatment. In the prospective study of Mueller et al. [17], 237 vertebrae in 98 patients were placed by 474 cement-augmented pedicle screws. Although no symptomatic cement leakage was observed, asymptomatic paravertebral cement leakage was seen in 88 patients and pulmonary cement embolism was found in 4 patients. Martín-Fernández et al. [26] reported 62.3% (650/1043 screws) ratio of cement leakage in 313 patients. Two of those patients had radicular pain, and 13 patients developed deep infections that had to be treated with revision surgeries. A total of 180 screws had to be removed in 56 patients. Those studies suggest that screw augmentation should only be performed when there is high probability of screw loosening. This makes it important to find a preoperative tool with high accuracy to predict the incidence of screw loosening.

In our clinical practice, we found that when the sacral bone is involved in rigid fixation, the probability of screw loosening can be significantly higher than cases with pedicle screw fixation of lumbar vertebra only. Therefore, it is especially important to find a predictive index for the screw loosening after the rigid fixation of the sacral bone. Quality of bone is the main contributor for the stability of pedicle screws because it decides the strength of screw bone interface. Due to decreased osseointegration at screw bone interface in patients with osteoporosis, they face higher risk of screw loosening after spinal surgeries. Therefore, it is plausible to use preoperative bone mineral density of the lumbar spine to predict the risk of screw loosening after spinal surgeries. It has been previously reported that CT-based Hounsfield units can be used to assess the quality of bone, which was also proven by many other authors [27–29].

By assessing the lumbar bone mineral density in routine using multidetector row CT, Schwaiger et al. found that in patients with lower Hounsfield units were more likely to experience screw loosening [30]. In the study of Bredow et al. [31], preoperative CT scans were used to assess the risk of pedicle screw loosening in 365 patients who received lumbar and thoracic spinal fusion surgeries. During a follow-up of 50.8 months, there were a total of 45 patients with screw loosening, whose CT-based overall vertebral mean bone density was 116.3 ± 53.5 HU, which was 132.7 ± 41.3 HU in patients with no screw loosening, indicating the predictive value of preoperative CT scan attenuation on postoperative screw loosening. Sakai et al. used the HU of screw trajectory to predict screw loosening after single-level spinal fusion surgeries in 52 patients with 206 screws, and HU of screw trajectory is an independent risk factor for screw loosening [32].

Although there were some reports on the correlation of HU value and the incidence of screw loosening in the lumbar spine, few studies were carried out to find HU-based criteria to predict sacral screw loosening. In the current study, we retrospectively analyzed the relations between Hounsfield units and the incidence of screw loosening after pedicle screw fixation in the sacral bone. In the current study, we measured the HU value of the sacral bone. Results of our study showed significant difference (*P* < 0.01) between the screw loosening group and control groups, indicating the correlation between low HU value of the sacral bone and the high incidence of screw loosening of the sacral bone, which was further proven by the Pearson correlation tests (*r* < 0.01). Area under the curve in ROC curve analysis was 0.674 (95% CI: 0.592-0.756), indicating relatively high diagnostic value of CT attenuation. Further analysis on the statistical data showed a potential cutoff value of 200 with the sensitivity of 64.8% and the specificity of 62.4%. Although a HU value of 200 suggests more than 60% chance of screw loosening, considering the potential fatal complications of cement augmentation and complexity of revision surgery in cases of screw loosening after cement augmentation, we propose a relatively mild approach such as expandable screws to increase the stability of screws when the CT attenuation value of the sacrum on the horizontal plane is lower than 200 HU. In the meanwhile, there was 90% sensitivity when the HU value is lower than 150; it may be plausible to use more radical methods such as bone cement augmentation to increase pullout strength and avoid screw loosening in those cases.

Considering the relatively small sample size and retrospective nature of the current study, more prospective studies with larger patient inclusion should be carried out to further test our conclusion. Besides the HU value of the sacral bone, the HU value of the lumbar spine could also provide valuable information on the bone mineral density and the possible of screw loosening after surgery, which should be further analyzed in future studies. Except from the HU value, there are other factors such as patient age, segments of internal fixation, overall health status, and the vigor of the patient. In the meanwhile, most of the patients with pedicle screw loosening did not show any symptoms and require further treatment. All those factors should be taken into consideration when deciding whether or not to apply screw augmentation and to use what type of screw augmentation technique in the patient.

## 5. Conclusion

Analyzing 200 patients with at least 12 months of follow-up, we propose 200 HU and 150 HU as cutoff points in the horizontal plane to take moderate and radical measures for screw augmentation to prevent screw loosening in the sacral bone.

## Figures and Tables

**Figure 1:** The region of interest (ROI) on the horizontal plane of the sacrum, and the radiologic attenuation was recorded in HU.

**Figure 2:** ROC curve analysis on the predictive validity of HU value of the sacrum.

**Table 1:** Demographic characteristics of the included patients in two groups.

	Nonloosening	Loosening	*P*
Male/female	63/28	51/20	0.43
Age	59.6 ± 7.5	66.2 ± 8.0	<0.01
Time of follow-up	18.2 ± 10.9	19.5 ± 12.3	0.48
BMI	24.8 ± 3.4	25.5 ± 3.9	0.23
Smoker	9	5	0.36
Diabetes	27	16	0.20
HU	225.8 ± 62.4	188.9 ± 54.6	<0.01

## Data Availability

The data is available from the corresponding author under reasonable request.
